# Application of Magnetic Resonance Diffusion Tensor Imaging in the Clinical Diagnosis of Disc Herniation after Lumbar Spine Injury

This article has been retracted.

**DOI:** 10.1155/2021/6610988

**Published:** 2021-03-10

**Authors:** Penghuan Wu, Chengyan Huang, Wenhu Li, Aidong Yuan, Anmin Jin

**Affiliations:** ^1^Department of Spinal Surgery, Zhujiang Hospital, Southern Medical University, Guangzhou, Guangdong 510282, China; ^2^Department of Orthopaedics, Affiliated Shaoguan First People's Hospital, Southern Medical University, Shaoguan, Guangdong 512000, China; ^3^Department of Radiology, Zhujiang Hospital, Southern Medical University, Guangzhou, Guangdong 510282, China

## Abstract

Magnetic resonance diffusion-weighted imaging (DTI) provides a unique perspective on the pathophysiological and microstructural changes during spinal cord injury, with high spatial specificity; meanwhile, NM reflects the conduction and integrity of neuroelectrical signals in spinal cord fiber tracts, with time-specific and dynamic evaluation effects. The fractional anisotropy (FA) value, SEP amplitude, and neurological function score or improvement rate are correlated. The combination of DTI and NM can more reliably quantify the spinal cord function, evaluate the effectiveness of treatment, and determine the patient's prognosis, which can provide reference for clinical decision making and future research for SCI patients. That is, the lower the preoperative FA value and the lower the SEP amplitude, the worse the preoperative and postoperative neurological function, the lower the improvement rate, and the worse the prognosis of patients. Therefore, we believe that spinal cord function can be graded according to JOA scores to find the corresponding FA and SEP amplitude ranges and that, by measuring FA and SEP amplitude in the future, we can reverse the assessment of spinal cord function, expected postoperative improvement, and long-term prognosis. At the same time, FA values can also help determine the nature of the lesion to some extent.

## 1. Introduction

DTI is an emerging imaging modality based on magnetic resonance diffusion-weighted imaging (DWI), which has a higher spatial resolution than NM and is better able to describe the pathophysiological changes in the spinal cord than conventional MRI, with histological correlation but almost zero temporal resolution [1]. By measuring data parameters and tracing the alignment of spinal tracts, DTI can complement traditional MRI and provide a more sensitive and intuitive description of spinal cord injury [2]. fMRI is another advanced MRI-based noninvasive examination technique that has not yet been widely used in clinical practice, but fMRI can be used to measure changes in blood flow and oxygenation around the metabolically active area, indirectly reflecting spinal cord function [3]. Conventional MRI is considered a reliable test for diagnosing spinal cord disease and guiding surgical access, but it has been well documented that lesions resulting in damage to the microstructure of the spinal cord sometimes cannot be demonstrated on conventional MRI [4]. DTI is a development and deepening of DWI, an examination modality based on the determination of the direction of movement of water molecules in the extracellular components of biopsies, which describes the attenuation of water molecules in the diffusion tensor field, reveals the connections between nerve cells, and enables noninvasive imaging of the spinal cord. DTI has long been used to determine the preoperative compression or infiltration of white matter fiber tracts in patients with brain tumors [5]. Currently, many animal models have suggested the correlation between DTI parameters and pathophysiological changes during recovery from spinal cord injury. Likewise, we have a reason to believe that DTI can provide accurate reference data for the diagnosis and treatment of patients with acute or chronic spinal cord injury [6].

DTI, as a special sequence of DWI and based on which computer software is used to trace white matter fiber tracts to form a fiber tract tractography (DTT), is currently the only method to noninvasively and clearly reconstruct nerve conduction tracts on living tissues, which has the sensitivity and sensitivity lacking in other imaging techniques [7]. DTI is a further development of DWI, where the dispersion tensor is not a flat process, but requires the application of gradient fields in multiple directions, at least six noncollinear directions of the dispersion-sensitive gradient directions, to provide a finer depiction of the tissue structure by quantifying the signal data of the anisotropy of the water molecule dispersion in 3D space [8]. The apparent diffusion coefficient (ADC) and the fractional anisotropy (FA) are two commonly used DTI parameters to quantify the dispersion or spatial displacement of water molecules, providing microscopic properties and pathological abnormalities of the tissue structure. DTI describes the shape and structure of spinal cord fiber tracts by quantifying the displacement of extracellular water molecules by the diffusion tensor. Unlike DWI, which describes “isotropic dispersion” (i.e., the degree of dispersion is not limited by direction), DTI describes “anisotropic dispersion,” which means that the water molecules disperse in all directions at varying distances [9]. In normal human tissue structures, water molecules are least restricted when their dispersion is oriented in the same direction as the nerve axons but are most restricted and slowest when they are vertical due to the presence of axonal myelin [10–14]. More precisely, this direction-dependent diffuse variability is referred to as “diffuse anisotropy” and is often quantified by the FA value, which, from 0 to 1, describes the anisotropy of different tissues. The FA of cerebrospinal fluid is infinitely close to 0, whereas the FA of white matter fiber tracts is infinitely close to 1 due to the high anisotropy [15]. It is because of this “anisotropy” that white matter fiber tract DTI imaging is possible. An increase in the extracellular gap (e.g., demyelination, axonal injury, and dispersion of white matter fiber tracts) and a decrease in the intracellular gap (e.g., edema) decrease the rate of axial dispersion of water molecules, ultimately leading to a decrease in the FA of the damaged spinal cord [16].

MR functional imaging and quantitative MR imaging of intervertebral discs have become hot topics of research in recent years. Normal intervertebral disc tissue is mainly composed of collagen fibers and proteoglycans, and degenerated disc tissue shows reduced water content, loss of proteoglycans, and fracture of collagen fibers, and these changes can be visualized in vivo by noninvasive MR functional imaging. MR diffusion-weighted imaging (DWI) or diffusion tensor imaging can quantify the diffusion capacity of water molecules in intervertebral disc tissue in three-dimensional space as shown in Figure 1. T2 values are influenced by the water content of the articular cartilage or disc, the proportion of proteoglycans, and the orientation of collagen fibers. The relationship between disc diffusion parameters and T2 relaxation time and the composition and tissue arrangement of the intervertebral disc tissue has been well documented. The method to study the function of intervertebral discs under intervertebral disc loading conditions, some domestic open magnetic field studies, and the author's previous studies through the use of homemade pedal load device to bear 40%–50% of its own body weight found that the loading condition can better simulate the pathophysiological characteristics of the intervertebral discs in the upright state; while nonloading intervertebral disc protrusion degree increases, the spinal canal area shrinks; short-term loading can affect mild degenerative discs diffusion function, the apparent diffusion coefficient is reduced, and the correlation between short-term load and T2 relaxation time, which reflects tissue composition, is not completely clear.

In recent years, several new and quantitative techniques for MRI have evolved and matured, including diffusion-weighted imaging (DWI), diffusion tensor imaging (DTI), magnetic resonance spectroscopy (MRI), and quantitative imaging (MRI). Resonance spectroscopy (MRS), T2 relaxation time, and T1*ρ* measurement have been applied in many fields and are now also used in the quantitative diagnosis of the biological microstructure and physiological state of vertebrae and intervertebral discs. Magnetic resonance diffusion-weighted imaging (DTI) provides a unique perspective on the pathophysiological and microstructural changes during spinal cord injury, with high spatial specificity; meanwhile, NM reflects the conduction and integrity of nerve signals in spinal cord fiber tracts, with time-specific and dynamic evaluation effects. The FA value, SEP amplitude, and neurological function score or improvement rate are correlated. By combining DTI and NM, spinal function can be quantitatively quantified, and the effectiveness of treatment is evaluated, and the patient's prognosis can be judged. This makes reference to the clinical decision-making and future study of the SCI patients. In other words, the preoperative FA level is lower and the amplitude of SEP is lower, and the preoperative and postoperative neurological function deteriorate, and the improvement rate is lowered, and the patient prognosis is deteriorated. Therefore, the spinal cord function is graded according to JOA score, and the corresponding FA and SEP amplitude range can be found, and it is possible to reverse the evaluation of the spinal function by measuring FA and SEP amplitudes in the future, and the postoperative improvement long-term prognosis can be expected. At the same time, the FA value also helps to determine the nature of the lesion to some extent.

## 2. Research Methods

### 2.1. Research Subjects

Twenty-five patients with lumbar intervertebral disc herniation treated with PTED, aged 20 to 60 years, average 43 years, 14 males and 11 females, were included in this study (Table 1). The duration of the disease (time from the first appearance of radicular pain or numbness in the lower extremities to the preoperative DTI scan) ranged from 2 to 13 months, with an average of 5 months. Inclusion criteria were (1) a single segmental medullary prominence compressing a single nerve root; (2) unilateral nerve root symptoms (pain or numbness); (3) patients undergoing MRI within the acceptable range of pain (some patients with severe pain were examined after conservative treatment); (4) surgery performed by the same physician. Exclusion criteria were multiple neurogenic lesions, history of lumbar and lower extremity surgery and trauma, and lumbar spinal stenosis. Most of the case-control cases confirm that the long-term surgical results of two procedures are equivalent. Minimally invasive pulmonuclear extraction, especially pted, is widely promoted because of the advantage of reducing soft tissue damage and postoperative complications. At present, the effectiveness of the lumbar disc herniation is evaluated mainly by the relaxation of the clinical symptoms and the periodical MRI examination, but there are some patients with clinical symptoms such as lower extremity pain and numbness, even if the appropriate pressure reduction of the compression nerve is indicated by the periodic MRI inspection. Root: it makes it difficult to evaluate efficacy and further treatment.

### 2.2. Research Methods

The same Siemens 3.0 TMRI scanner was used preoperatively and in March postoperatively. AXI T1-VIBE anatomical positioning and AXI SE-EPI DTI scanning were performed after routine MRI scanning. DTI scan parameters are TR/TE 7 500/95 ms, layer thickness/spacing 3/0 mm, FOV 230 × 230 mm, MPG 20 directions, b-value (0, 800 s/mm^2^), and scan time 8 min12 s. The scan range is from the inferior border of the T3 vertebral body to the S1 vertebral body. Fiber tracing, FA, and ADC values were determined using Siemens workstation Neuro 3D software. The preoperative and postoperative DTI parameters were determined in conjunction with the AXI T1-VIBE anatomical positioning images to ensure that the two measurements were as consistent as possible. The regions of interest (ROIs) were measured three times consecutively and averaged at three levels, from the nerve root compression to the distal level. To avoid partial volume effects, the ROIs were limited to 25 to 50 mm^2^.

### 2.3. Statistical Analysis

SPSS 20.0 statistical analysis software was used for the comparison of preoperative and postoperative data. Paired-sample *t*-test was used for preoperative and postoperative data comparison, and independent-sample *t*-test was used for bilateral nerve root data comparison. Pearson's correlation analysis was performed to test the correlation between DTI parameters and disease course. *P* < 0.05 was considered statistically significant. At present, traditional open-window nucleus pulposus extraction and minimally invasive nucleus pulposus extraction are the main clinical procedures for the treatment of lumbar intervertebral disc herniation. The majority of case-control cases confirm that the long-term surgical results of the two procedures are comparable. Minimally invasive nucleus pulposus extraction, especially PTED, has been widely promoted because of its advantages of reducing soft tissue injury and postoperative complications. Currently, postoperative efficacy of lumbar intervertebral disc herniation is mostly evaluated by the relief of postoperative clinical symptoms and routine MRI examination, but some patients still have clinical symptoms such as lower limb pain and numbness even though routine MRI examination shows adequate decompression of the compressed nerve root, which makes it difficult to evaluate the efficacy and further treatment. It is believed that the improvement of the microstructure of the compressed nerve root and the relief of the surrounding inflammatory response is the key to the success of treatment.

DTI is an effective method for noninvasive tracing of nerve fiber tracts and for quantitative assessment of nerve injury. Most of the literature confirms that the FA and ADC values of DTI can quantify the microstructural changes of compressed nerve roots in lumbar intervertebral disc herniation, with decreased FA reflecting tissue damage, demyelination, and axonal defect of the compressed nerve root, and increased ADC associated with inflammatory response and tissue edema. In a study of 13 patients with lumbar intervertebral disc herniation of an average duration of 38 days, it was found that the FA value of the compressed nerve root at 6 months after surgery was significantly higher than that before surgery, but it was not mentioned whether there was a difference in FA value between the affected and healthy side after surgery. It was found that the FA value of the compressed nerve root in the first month after surgery was higher than the preoperative value, and there was no statistically significant difference in the FA values of the bilateral nerve roots after surgery, but the preoperative duration of the disease was not provided. The results of the present study showed that the FA value of the affected nerve roots was higher after surgery than before, which is consistent with the results of the previous authors' study. However, in this study, the FA value of the affected nerve root was still lower than that of the healthy side, and the difference between the FA value of the stressed nerve root before and after surgery showed a significant negative correlation with the duration of the disease, so the duration of the disease may affect the recovery of the stressed nerve root structure after surgery.

## 3. Magnetic Resonance Imaging to Evaluate the Relationship of Intervertebral Disc Degeneration

### 3.1. Spinal Vertebral Structural Changes in Patients with AIS

Vertebral body rotation and wedge deformity are the main manifestations of scoliosis, as shown in Figure 2, and histological studies have shown histological differences between the concave and convex structures of the vertebral body with wedge deformity. Following the Hueter-Volkmann law, compressive stresses during vertebral body growth inhibit growth of the vertebral body growth plates, and therefore, the cartilage of the concave end plate thins. Due to the remodeling function of the bony structure, the trabecular bone in the vertebral body rebuilds when the pressure increases, resulting in an increase in bone mass and a stronger bone structure, and decreases when the pressure decreases [17]. Animal studies have shown that, during the dynamic growth of scoliosis vertebrae, the concave side of the vertebral body overgrows and there is a continuous migration of bone volume from the convex to the concave side of the vertebral body to resist the increased compressive stress on the concave side of the vertebral body. Animal studies have also shown that the convex side of the vertebral body in AIS patients has a thinner bone cortex, thinner trabeculae, and wider trabecular gaps, while the concave side has a thicker bone cortex, thicker trabeculae, and smaller trabecular gaps. Previous work [18] reported that the cancellous bone of the vertebral body is more porous on the convex side than the concave side, and the cortical bone of the convex side is thinner than the concave side. High-resolution peripheral quantitative computed tomography (HR-p QCT) observed fewer trabeculae and greater trabecular spacing in the distal radius of girls with AIS, indicating an abnormal bone structure and stress index in patients with AIS [19–23]. In conclusion, the microstructural changes present in the vertebral bodies of scoliosis patients include reduced bone volume compared to normal vertebrae and differences in the microstructure of the bone on the convex side of the vertebral body. Reduced bone mass is common in patients with AIS and is presumed to be associated with abnormal bone metabolism. The vicious cycle theory suggests that asymmetric growth of the vertebral body leading to asymmetric stresses on both sides of the spine will exacerbate the microstructural changes in the vertebral body and that the two factors will interact during spinal growth to form a vicious cycle that will exacerbate the progression of scoliosis. Early diagnosis can assist in early intervention, thereby alleviating the progression of scoliosis, reducing labor and loss of life, and improving patient prognosis.

### 3.2. Magnetic Resonance Diffusion Imaging of Vertebral Structures

Magnetic resonance imaging is a radiation-free imaging modality that is increasingly being used in the skeletal system. Conventional MR images, including T1- and T2-weighted images, are good for assessing spinal morphological abnormalities in AIS but do not provide any quantitative information about the microstructure of the vertebral body. DWI is able to assess microstructural changes in trabecular tissue by using the apparent diffusion coefficient (ADC) value. A more advanced diffusion imaging technique, DTI, assesses differences in the restricted diffusion of water molecules within the tissue based on mean diffusion (MD) values, while fractional anisotropy (FA) values emphasize differences in water molecules within porous bone [24]. Anisotropy of diffusion: cancellous bone causes compression fractures in vertebrae with the lowest ADC values and highest FA values, and fiber beam imaging directly demonstrates the presence of blue fibers in compression fracture vertebrae with preferential diffusion in a cephalocaudal direction, and the preferential diffusion of water molecules in cancellous bone in a cephalocaudal direction may be closely related to the altered trabecular arrangement of bone in collapsed fracture vertebrae.  Figure 3 shows the anisotropy of the cancellous bone in the vertebral body. The changes in the mechanical behavior of the cancellous bone following the tested mechanical directions suggest that the anisotropy of the bone stresses is characterized by the anisotropy of the bone trabeculae and the preferential orientation of the trabeculae and that the anisotropy is influenced by both the preferential orientation force acting on the bone and the resistance force, i.e., the force acting on the bone and the reaction force of the bone constructing the anisotropy. The study also shows that the stress characteristics of cancellous bone depend on the anisotropy of the bone density and trabecular structure and that the cancellous bone is ordered along the main stress direction to avoid shear forces on the trabeculae, while minimizing the bending moment and placing the trabeculae in a favorable mechanical state where the axial forces are dominant. Diffusion tensor imaging revealed the presence of parallel aligned tensor fibers in the epiphysis and adjacent symphysis of long bones, and these structures were directly revealed by the computational method of tracing fiber bundles. Previous studies have used DTI to assess potential abnormalities in the spinal cord of patients with AIS.

The cancellous bone of the vertebral body is composed of trabecular bone and bone marrow, which is composed of fat and water. Almost all of the water in the vertebral body comes from the red bone marrow, which gradually decreases with age and increases with fat content. Hydrogen proton spectroscopy (1H-MRS) allows quantitative analysis of the bone composition, especially the fat and water content, as shown in Figure 4. The vertebral body spectral signal is composed of two main components: a water signal produced by the red bone marrow, red lineage cells, and lymphocytes, and a fat signal produced by adipocytes. 1H-MRS commonly used measurement parameters include fat content (fat fraction%, FF%), LWR (lipid water ratio, LWR), and line width (FF% = LWR/(LWR + 1) × 100%, LWR = water peak/fat peak, peak height around 4.65 ppm is water peak, and peak height around 1.3 ppm is fat peak (ppm indicates 10–6). Full width at half-maximum (FWHM), expressed in Hz, was related to the compound's T2^∗^ value and magnetic field uniformity, which influenced the water and fat peaks. By measuring FF% in the lumbar vertebrae of healthy volunteers and correlating it with age and gender, it was concluded that FF% increased linearly with age and that there was a gender difference, with women having less fat in the vertebrae than men. It was found that LWR was positively correlated with age and negatively correlated with BMD; LW was correlated with intravertebral fat content and BMD but was greatly influenced by the inhomogeneity of the magnetic field generated by the trabecular bone. The results suggest that neither the water peak nor the fat peak LW is significantly related to age, whereas the former suggested that the water peak LW narrows with age. Osteoporosis is the most common clinical disease of bone metabolism and is characterized by decreased bone density, increased brittleness, and susceptibility to low-energy fractures. With age, the vertebral body hematopoietic tissue decreases, trabecular atrophy decreases, the trabecular space increases, fatty tissue increases, and the yellow bone marrow fills the widened trabecular space. It has been shown that vertebral FF% increases in patients with osteoporosis, with increased fat content in the bone marrow, decreased cancellous bone content, and decreased BMD, speculating that FF% may be used directly to assess bone density. We measured LWR and FF% in the lumbar vertebral bodies of women in the youth and middle-aged and elderly groups. Some work has been done on the 1H-MRS technique in the study of vertebral body lesions, but there are still some problems, including motion artifacts and poor reproducibility due to long scan times.

### 3.3. Intervertebral Disc Structural Changes in Idiopathic Scoliosis

The intervertebral disc, as the connecting structure between the vertebral bodies, accounts for approximately one-third of the total length of the spine, and the growth of the intervertebral disc and the end plate is the factor most directly related to the growth of the spine. Some scholars believe that changes in the composition and structure of the intervertebral discs and end plates are the cause of the development of scoliosis and that biomechanical abnormalities of the spine in scoliosis patients can lead to changes in the structure and composition of the intervertebral discs. It has been suggested that, during the rapid growth of children with scoliosis, disc wedge changes occur first, followed by progressive wedge changes in the vertebral body. Through the observation of 37 cases of adolescent scoliosis patients with vertebral body and disc wedge changes, it was found that the degree of vertebral body and disc wedge changes increases with the progression of scoliosis, and it is believed that the abnormal growth of the cartilaginous end plates of the vertebral body may be the main cause of vertebral body wedge changes. Using the simplified model matrix method, we deduced that the imbalance in the arrangement of the fibrous crystals in the fibrous annulus is the cause of scoliosis progression. Previous authors have observed degeneration-related microstructural changes in the intervertebral discs of scoliosis patients, including disorganization of the elastic fibrous reticulum of the intervertebral disc annulus and clustered cell mass structure, whereas these degenerative microstructural changes were absent in the discs of age-matched healthy controls. It has been suggested that abnormal mechanical stresses can accelerate disc degeneration. The reduced proteoglycan and water molecule content in the discs of patients with scoliosis compared to normal discs was found to be an important pathological change in early disc degeneration. Intervertebral discs play a key role in the maintenance of spinal flexibility in scoliosis patients, and preoperative flexibility assessment is an indicator of the patient's trunk deformity and intraoperative fusion of segments, which can provide reference for preoperative planning and help predict the degree of postoperative orthopedic deformity.

Biologic therapies such as genetic, cellular, or growth factor-based therapies can repair degenerated discs to some extent and prevent further progression of the degeneration, so early diagnosis and evaluation of disc degeneration are helpful for early intervention and prognosis of scoliosis patients. However, routine MRI is not sensitive to early degeneration of discs, and the morphology and signal of discs that have already undergone histological degenerative structural changes do not change significantly on T2WI. In recent years, some scholars have used MRI to study the distribution of T2 signal intensity in the nucleus pulposus region of scoliosis patients and found that there is a difference in the distribution of T2 signal intensity in the nucleus pulposus region of scoliosis patients, and this difference correlates with the pathological changes and severity of disc degeneration. Prediction: it can be used as a supplement to the existing diagnostic tools, so it is recommended as an early biological marker of disc degeneration and can be used in the prognosis of scoliosis and in the selection of treatment methods. The advent of multiple new MR techniques, including DWI, DTI, T2 relaxation time, and T1*ρ* measurements, has been applied in the diagnosis and quantitative evaluation of early disc degeneration.

## 4. Results and Discussion

Both DWI and DTI are diffusion imaging and are the only instruments that can noninvasively observe the microscopic diffusion motion of water molecules in living tissues, DWI reflects the restricted motion of water molecules by measuring the ADC value, and DTI is an advanced form of diffusion imaging that allows a more accurate description of water molecules in tissues by applying diffusion sensitive gradients in multiple directions to measure the degree and direction of diffusion. The MD value emphasizes the difference in the restricted diffusion of water molecules within the tissue, while the FA value emphasizes the anisotropy of water molecule diffusion within the tissue. The periphery of the intervertebral disc is a fibrous ring structure, which is formed by the cross-arrangement of fibrous crystals, and the dispersion of water molecules is restricted to the direction consistent with the direction of the fibers. T2 relaxation time (i.e., T2 value) is the constant of T2WI signal decay, which is related to the content of proteoglycans, collagen, water, and other molecules in the tissue. Changes in molecular content: animal studies were performed on 35 rabbit lumbar intervertebral discs, and it was confirmed that T2 relaxation time was significantly correlated with the expression of proteoglycans and type II collagen in the nucleus pulposus of the intervertebral discs, that T2 mapping was sensitive to disc degeneration, and that T2 values and T2 mapping could achieve in vivo understanding of the pathophysiology of disc degeneration. T2 mapping was performed on the intervertebral discs of 37 asymptomatic volunteers, and T2 values and Pfirrmann grades were correlated, as shown in Figure 5, which showed that there was age-related degeneration of the intervertebral discs and that the T2 relaxation time of the nucleus pulposus decreased with increasing Pfirrmann grade. T2 mapping was performed on 30 obese simplex and 30 normal-weight healthy volunteers, and it was confirmed that T2 mapping could detect biochemical changes in the early stages of lumbar disc degeneration and that obesity may accelerate the degeneration of the disc.

T1ρ imaging, which is the spin lattice time within the rotating frame, is sensitive to low-frequency motion and can be used to probe the slow motion of free water molecules on the surface of macromolecules; thus, T1ρ imaging values can be used to assess the proteoglycan content of intervertebral disc tissue. We believe that T1ρ values are sensitive to early changes in proteoglycan and water content in the lumbar intervertebral disc. MR multiparametric imaging studies of 13 AIS patients showed that the parietal intervertebral disc was more prone to degeneration than the distal intervertebral disc, T1ρ values were reduced, and the degree of disc degeneration was significantly correlated with Cobb's angle, as shown in Figure 6. The relationship between water and proteoglycan peak area ratio, T1ρ value, and Pfirrmann score was evaluated by quantifying the water and proteoglycan content of the intervertebral discs using MRS. The results showed that the peak area ratio of water to proteoglycan was significantly increased during disc degeneration, and the disc T1ρ value was significantly correlated with proteoglycan loss, but not with water content. It is believed that T1ρ imaging can be used as a biological marker of early disc degeneration.

DTI parameter values can indicate the degree of damage to the white matter fiber tract. We performed DTI examination and later DTT reconstruction on 15 patients with spinal cord compression. The results showed that FA decreased in 10 patients and ADC increased in 2 patients. We also performed DTI on 5 patients with low-grade spinal cord astrocytoma and 10 healthy volunteers, and the results showed that the FA values at the tumor sites were decreased, and DTT was applied to reconstruct the posterior and lateral tracts of the corticospinal cord, showing that the spinal cord tracts of the healthy volunteers were normal and complete, while the white matter tracts of the patients were deformed and broken. However, they also found that white matter fiber tract tracking was more effective in solid tumors and less sensitive in cystic tumors. Compared to solid tumors, the increased diffusion of water molecules leads to larger errors and poorer accuracy of DTI parameters in cystic tumors or other tumors with extremely severe peritumoral edema. In addition, some authors have reported increased FA values in the damaged spinal cord in some patients. We have reported an increased FA in the lesion area of the spinal cord in a patient with spinal astrocytoma. This phenomenon was considered to be related to two conditions: first, severe peritumoral edema leading to the transfer of extracellular water into the intracellular space and, second, shrinkage of the extracellular environment due to cell permeability in an inflammatory environment. Although this theory has not been fully tested, it may be related to the encapsulation, invasion, and infiltration of the spinal cord by astrocytomas. The data obtained from DTI for white matter fiber imaging, or DTT, is a further development of the DTI technique, which allows identification of white matter fiber channels and their interconnections, observation of the direction of travel of spinal cord fiber bundles, and confirmation of tumor boundaries with surrounding tissues, providing an image and data basis for surgical planning. In early cases of children with intramedullary tumors, it has been demonstrated that the displacement or infiltration of fiber tracts in DTI and DTT images is decisive for the choice of surgical approach. A total of 10 patients (8 males and 2 females) between the ages of 8 and 12 years were enrolled in the study and underwent surgical treatment. 8 patients had significant DTI and DTT migration of the spinal cord fiber tracts, 7 of whom underwent total tumor resection and one of whom underwent near-total tumor resection. 2 patients showed significant invasion of the spinal cord. The other two patients showed significant spinal cord infiltration and only underwent pathologic biopsy.

This study shows, as shown in Figure 7, that when DTI indicates that the tumor's effect on the spinal cord is mainly compressional excursion, a clear peritumor border can be found intraoperatively to achieve total resection of the tumor with a good prognosis; however, when the tumor is mainly infiltrating the spinal cord, partial resection with decompressive nature and biopsy may be more recommended. Results also show that DTI has a sensitivity of 87.5% for predicting tumor resectability, with a specificity of 100%, a positive prediction rate of 100%, and a negative prediction rate of 83.3%; DTI can predict tumor resectability and guide the best surgical approach and method and bring better prognosis for spinal cord tumor patients. The maximum resection of the vertebral body and intervertebral disc and the maximum preservation of the function of the spinal fiber bundle are also possible. In summary, scoliosis in AIS patients is associated with visible changes in the vertebral body and intervertebral disc wedge deformities, as well as changes in the microstructure and histological composition of the vertebral body and intervertebral discs. It plays an important role in both prediction and follow-up of treatment effects.

## 5. Conclusion

Magnetic resonance diffusion-weighted imaging (DTI) provides a unique perspective on the pathophysiological and microstructural changes during spinal cord injury, with high spatial specificity; meanwhile, NM reflects the conduction and integrity of neuroelectrical signals in spinal cord fiber tracts, with time-specific and dynamic evaluation effects. The FA value, SEP amplitude, and neurological function score or improvement rate are correlated. The combination of DTI and NM can more reliably quantify the spinal cord function, evaluate the effectiveness of treatment, and determine the patient's prognosis, which can provide reference for clinical decision making and future research for SCI patients. That is, the lower the preoperative FA value and the lower the SEP amplitude, the worse the preoperative and postoperative neurological function, the lower the improvement rate, and the worse the prognosis of patients. Therefore, we believe that spinal cord function can be graded according to JOA scores to find the corresponding FA and SEP amplitude ranges, and by measuring FA and SEP amplitude in the future, we can reverse the assessment of spinal cord function, expected postoperative improvement, and long-term prognosis. At the same time, FA values can also help determine the nature of the lesion to some extent.

## Figures and Tables

**Figure 1:** Quantitative analysis of dispersion tensor imaging in 3D space.

**Figure 2:** Histological study of the concave and convex structures of the vertebral body in wedge variation.

**Figure 3:** Changes in the mechanical behavior of cancellous bone.

**Figure 4:** 1H-MRS for quantitative analysis of osteoporosis.

**Figure 5:** Correlation of T2 mapping on disc degeneration.

**Figure 6:** Correlation between the degree of disc degeneration and Cobb's angle.

**Figure 7:** Patient DTI analysis results.

**Table 1:** The general information of selected patients.

Group	Average age (years old)	Gender (male/female)	Course of disease (month)	Injury part	
				Left	Right
Control	20–60	14/11	2–13	18	22
Observation	20–60	14/11	2–13	18	22

## Data Availability

The data used to support the findings of this study are available from the corresponding author upon request.
